The article "Progress and Emotion Expression of Campus Cultural Innovation Goods Based on Data Mining under Culture Shock Environment" was retracted in 2023. Reasons: signs of a paper mill; suspected computer-generated content; unreliable results or conclusions; concerns about the data.

# Progress and Emotion Expression of Campus Cultural Innovation Goods Based on Data Mining under Culture Shock Environment

**DOI:** 10.1155/2022/4874748

**Published:** 2022-09-12

**Authors:** Liyuan Zhang

**Affiliations:** Yan'an University, Yan'an, Shanxi 716000, China

## Abstract

With the rapid progress of economy and globalization, the characteristic culture of universities is inevitably eroded by the strong mainstream culture from outside. The best way to maintain culture is to turn it into goods. Productization can make culture vivid and vivid and circulate in use. Universities are the carrier of education and the progress of excellent culture. Campus culture refers to all tangible and intangible objective existence created artificially and formed for a long time in a specific school environment, which can deeply reflect the characteristics of the school. This article proposes an optimized design scheme for the progress and emotional expression research of campus cultural innovative goods in universities. It constructs the graphics recognition of campus cultural goods through the data mining system and then focuses on the problem of graphics recognition based on DL (deep learning). An enhanced DL model and arithmetic are proposed to enhance the accuracy and efficiency of graphics recognition. Finally, the simulation test and analysis are carried out. The simulation results show that the proposed arithmetic has certain accuracy, which is 10.23% higher than the traditional DL arithmetic. Campus culture can also play a powerful role in emotional edification and personality shaping for teachers, students, and campus workers. Excellent cultural and innovative goods can inherit the history, culture, and spirit of universities and can directly reflect the cultural heritage, characteristics, and graphics of universities. In addition to promoting the precipitation and inheritance of the long history and culture of universities and the spirit of the times, they can also strengthen the cultural exchange and spiritual communication among college level, alumni, teachers, and students, and people from all walks of life in universities, so as to actively promote the cultural and spiritual construction of universities.

## 1. Introduction

With the progress of social and cultural construction, the relevant departments of the state pay more and more attention to the cultural inheritance of universities. At present, it is mainly driven by cultural creativity with new thinking, new methods, and new influences as the core [1]. In particular, the national key universities pay special attention to the cultural and innovative goods of their own universities, mainly because these campus element goods spread the brand of the university and affect the feelings of teachers and students towards the alma mater [2]. The national policy has repeatedly stressed the need to strengthen the construction of national cultural soft power. The university campus is the base for breeding culture, and the campus teachers and students are the promoters and contributors of national cultural construction [3]. Therefore, the construction of campus culture in universities is also an important part of improving the soft power of national culture [4]. Secondly, for universities themselves, campus culture is a unique spiritual symbol of the campus. In recent years, universities have gradually designed their own cultural and innovative souvenirs based on campus culture and relying on campus characteristic culture. Consumer items that propagate ideas, symbols, and lifestyles are referred to as cultural goods. They can enlighten and amuse, helping to forge communal identity and shape cultural behavior. The school's symbols and academic philosophies serve as the foundation for the campus' cultural commodities. They have particular cultural meanings that help foster and create a positive campus cultural ambiance while also increasing the students' sense of cultural identification and togetherness. Teachers, students, and alumni feel strongly connected to one another thanks to campus culture. They are glad to disseminate campus culture through their work and studies and employ new and cultural campus products, which is great for the long-term development of the university cultural business. The development of campus culturally creative items can not only encourage the dissemination and interchange of campus culture, but it can also have some positive economic effects and increase the school's revenue. A worthwhile and insightful study was conducted based on the distinctive university culture.

The most basic elements of culture and emotion are symbols, and cultural symbols directly reflect the internal details of cultural and innovative goods [5]. Cultural symbol is a kind of mark, and its mark has uniqueness, regionality, and identification [6]. It is more dependent on the external environment of the generated cultural connotation and details [7]. Instead, the product is used as a communication medium to express specific cultural and emotional symbols, and to express the personalization of the product and the transmission of spiritual culture. This is the importance of the communication of cultural and emotional symbols [8]. In the design of cultural and innovative goods on campus, we should deeply explore the cultural feelings and emotional cognition that need to be spread on campus. “Campus environment, campus culture, and campus spirit” are the core elements that affect cultural emotional symbols. In the design process of cultural and innovative goods, users can have a certain emotional cognition through the transfer of the process, shape, material, and other aspects of the product itself. A unique neural network model is the DL model. DL has been used successfully in a variety of domains, including computer vision, speech recognition, natural language processing, and internet advertising. Since the DL Renaissance, it has been included into the most cutting-edge systems across a variety of fields, particularly in computer vision and automatic speech recognition. On frequently used datasets for evaluation, such as TIMIT (ASR) and MNIST (graphics classification), and a number of big vocabulary speech recognition tasks, new DL algorithms have been regularly improved and verified [9]. According to the outcomes, DL has a good capacity for learning and performs admirably. broad coverage and flexible design. Since DL neural networks contain numerous floors and a large breadth and may theoretically be mapped to any function, they are capable of handling highly challenging issues. Data is DL's primary resource, and the more data it has, the better it works. It is notably prevalent in the NLP, facial recognition, and graphics recognition domains. In view of the advantages of DL, this article adopts the convolution neural network graphics extraction method in DL to reduce the execution cost of the arithmetic. Through practice, it has been proved that this combination can not only reduce the calculation time but also enhance the quality and efficiency of the progress of cultural and innovative goods and the optimization of emotional expression on campus.

Campus cultural and innovative goods are very important in the process of improving and spreading campus culture [10]. On the one hand, the campus spirit and campus stories contained in the innovative goods of campus culture can arouse the resonance of students, enhance the sense of belonging and identity of teachers and students to campus culture, inject fresh blood into the construction of campus culture, and promote the formation of a good campus cultural atmosphere. On the contrary, the profound campus culture provides material with profound cultural connotation for the design of campus cultural and innovative goods, and provides material support for the design of campus cultural and innovative goods [11]. On the other hand, as a medium to spread campus culture, campus cultural, and innovative goods can help more people feel and understand campus culture, make them more eager to buy campus cultural and innovative goods, and provide economic guarantee for the progress of campus cultural and innovative industries [12].

In this article, the visual feature reconstruction model of the graphics of the progress and emotional expression optimization design of university campus cultural innovative goods is established. The template matching in the process of the visual reconstruction of the graphics of the product progress and emotional expression optimization design is carried out through data mining technology, and then, the fuzzy feature quantity of the graphics of the progress and emotional expression optimization design of university campus cultural innovative goods is extracted by CNN arithmetic. Its innovation lies in the following: (1) in this article, the convolution neural network graphic extraction method in DL is used to reduce the execution cost of the arithmetic. (2) This article constructs the key feature quantity of the graphics for the progress of cultural innovative goods and the optimal design of emotional expression on the campus of universities, and uses data mining technology to realize the product progress and the optimal design and identification of emotional expression.

## 2. Related Work

On the basis of campus culture, the innovative goods of campus culture are used as the media to stimulate the youth memory of more people, promote the design enthusiasm of the public, and drive the growth of campus innovative economy [13]. Excellent cultural and innovative goods can be used as communication carriers between schools, as a bridge to deepen the feelings between students and their alma mater, and also as a publicity channel for schools to face the society, so that more people are willing to understand the campus culture of Lanzhou campus [14].

Shaw et al. explained that “any product or combination of goods produced in the cultural and innovative industry, from the perspective of the final form of goods, cultural, and innovative goods include two interdependent parts: cultural and innovative content and hardware carrier.” Cultural and innovative goods are goods that add the core of culture on the basis of goods. They are goods with goods as the cornerstone and innovative design as the core. Both are indispensable and complement each other. Lee et al. analyzed the scale of Taiwan's existing cultural industries and the well-known cultural and innovative industrial parks throughout Taiwan. For example, Huashan cultural and innovative park, a demonstration base of Taiwan's cultural and innovative industries, Songshan cultural and innovative industrial park in Taipei, and Taiwan Chinese innovative park, all of these cultural and innovative industrial parks have the characteristics of “reusing idle plants”. For example, the predecessor of Songshan cultural and innovative park is Songshan Tobacco Factory. These cultural and innovative industrial parks have achieved innovative progress in the field of cultural and innovative industries by using their own historical background and characteristics and combining traditional process concepts [15]. Zhang and Wang believe that it is necessary to combine innovative ideas and experiential design, that is, what the audience needs is not only the beauty of the product itself but also the emotional design concept, so as to enhance the interaction between the product and the user, so as to meet the psychological satisfaction of the user [16]. Ucar analyzed the extraction methods and moral sources of many series of Chinese innovative goods of Taiwan Normal University with examples [17]. In the investigation and analysis of cultural and innovative goods in universities, Wang and Jian believe that they should have “artistic appearance, functional experience and cultural connotation reflection.” It is necessary to conduct a detailed analysis on the consumption groups, consumption demands, and other aspects of campus cultural and innovative goods to obtain data such as the consumption range of cultural and innovative goods and the portraits of consumer groups [18]. Christiaan studied the three levels of design: “instinctive, behavioral, and reflective.” From the perspective of campus cultural and innovative goods design and Norman's analysis, the design of campus cultural and innovative goods can be interpreted as three levels: direct application, concrete transformation design, and sublimation of freehand design. From this theory, we can more clearly judge the level and height of cultural and innovative goods [19]. Yuan et al. systematically explained the innovative industry and innovative management methods from the germination of creativity. Through the display of various cases, they analyzed the design process of individuals and teams in the innovative industry, and extended to innovative marketing and management methods, which is very worth reading [20]. Montalto et al. pointed out that in recent years, cultural and innovative industries around the world are booming under the guidance of relevant policies, extending to all aspects of life. It can be said that there are cultural creativity and business opportunities everywhere. With the progress and upgrading of schools, the issuance of campus cultural and innovative goods has become a key step in the construction of campus culture of universities around the world. The progress of campus cultural and innovative goods can not only expand the popularity of schools but also create new cultural and economic values [21].

There are few studies on the cultural and innovative goods of universities. There are no books that are suitable for the collection and records of the institute of cultural and innovative goods of universities. There is no perfect progress and management system of cultural and innovative goods. The cultural and innovative goods of universities are still in the initial stage of independent progress, unbalanced progress and immature. This article proposes an optimized design scheme for the progress and emotional expression research of cultural and innovative goods on campus. It extracts the graphics of cultural and innovative goods through data mining technology and then uses DL arithmetic to classify and identify the graphics. It optimizes the design of innovative goods from the aspects of campus cultural elements and cultural connotation, so as to make the product design more novel and unique.

## 3. Methodology

### 3.1. Build an Graphic Data Mining System to Analyze Cultural and Innovative Goods

The key to product Emotionalization lies in the communication between product functions and users' emotions to meet their psychological needs [22]. Psychologically speaking, human beings have many potential emotional needs, such as curiosity, performance, and desire. Therefore, attention should be paid to the matching between the user's nature and the emotional design of the product. The connotation of excellent emotional design requires the user to experience the product floor by floor in the use process. The cultural and innovative goods of universities carry the campus culture. Their form, semantics, and usage reflect the aesthetic principles and cultural and emotional connotation that match the product category and are committed to the campus users to obtain a happy emotional experience. Through the promotion of cultural and innovative goods, the cultural concept supported by the mainstream social standards can be transmitted to users, which can cause resonance and enable users to constantly enhance and enhance themselves under the cultural identity. This process is the emotional communication between users and goods. This interaction provides a shortcut for the spread of campus culture, which is the significance of emotional design.

The design of campus cultural goods should be based on graphics, through what we have seen and heard, and express the design concept and design emotion in kind. Image data mining system is required to automatically extract useful semantic information from graphics data. Image data mining is a technique used to mine the knowledge implicit in large-scale graphics data, the relationships within or between graphics, and various other patterns hidden in graphics data. In other words, graphics mining is to extract the implicit knowledge, the relationship between graphics data or other implicit patterns from the graphics database. Image mining has become the focus of attention. The realization of graphics data mining needs to be realized by computer vision, graphics processing, graphics retrieval, data mining, machine learning, database, and artificial intelligence.

Early graphics mining research concentrated on recommending an appropriate framework for carrying out the task. It is not possible to directly use a graphics database with original graphics data for mining. For the high-level mining model to be able to utilize the information, the original visuals must first be processed. Because it must leverage a variety of technologies—from graphics retrieval and indexing to data mining and pattern recognition—graphics mining systems are frequently difficult. A competent graphics mining system may produce knowledge and patterns beneath the graphics and give users efficient access to the graphics warehouse. Such a system typically has the following capabilities for this purpose: storage of graphics, processing of graphics, feature extraction, graphics indexing and retrieval, and pattern and knowledge finding. There are now two types of frames for graphics mining systems: function-driven and information-driven frames. The majority of the currently used graphics mining solutions operate within a function driven architecture. These systems are tailored and application-focused, and the framework is set up in accordance with the model's intended use. This paper suggests a target recognition-based paradigm for graphics mining. Target recognition is the foundation for image mining. The probable relationship between the targets and the background should be discovered. The second step of target recognition can be completed using the discovered potential relationship. The graphics mining framework is shown in Figure 1.

After graphics data mining, the data is preprocessed.

Data normalization (After data integration and combination, the intensity of each collected diffraction point may have systematic changes caused by various measurement errors and various physical factors, and the data processing process is required. First, the same diffraction point may be collected many times; secondly, theoretically, the diffraction intensity of a group of diffraction points connected by symmetry should be the same. The experimental measured values of these points with the same diffraction intensity in theory should be statistically averaged and supplemented with correction for radiation damage and absorption).

#### 3.1.1. Simple Zoom

Simple scaling's goal is to change the value of each data dimension, which may or may not be independent of one another, so that the final data vector falls inside a predetermined range, such as [0, 1] (depending on the data situation). In order to reduce the huge prediction error brought on by the large order of magnitude difference between the input and output data, the order of magnitude difference between the data for each dimension will be eliminated. Other techniques apply a linear transformation to the initial data, such as the minimal maximum method:

(1) $$\begin{array}{c} x^{*}=\frac{x-x_{\min}}{x_{\max}-x_{\min}}. \end{array}$$

#### 3.1.2. Sample-by-Sample Mean Subtraction

If the sample data is stable, that is, the statistics of each dimension of the data are subject to the same distribution, then it can be considered to subtract the statistical average value of the data from each sample for normalization.

#### 3.1.3. Feature Standardization

Feature normalization refers to (independently) making each dimension of data have a transformation with a mean of zero and a variance of 1. This normalization method is one of the most common methods.

### 3.2. Identification and Optimization of Cultural Creativity Based on DL

Human beings are symbolic animals. For example, goods with bright colors and beautiful shapes but no symbol rhythm cannot fully allow designers to fully express their inner feelings and thoughts through goods. It is through the purchase and use of the product that the user can have certain thinking interaction and emotional cognition with the designer through the symbol of the product. The cultural emotional symbols and the real value of goods are derived from a specific environment and cultural connotation, which is like a soul.

Image recognition is the process of employing computer technology to gather, process, and identify the target in the graphics. The most significant area of research in the subject of graphics recognition is the use of computers to recognize objects in graphics. DL emerged from the study of neural networks as one of the key research areas in the field of artificial intelligence. It creates a model with multiple levels and automatically extracts feature information from the low level to the high level, extracts features from the input data floor by floor, and generates more abstract and conceptual feature representations, simulating the process of how human brain neural networks process information. According on the structure and method of technology application, DL may be separated into three categories: generative depth structure, discriminant depth structure, and hybrid depth structure.

#### 3.2.1. Generative Depth Structure

The generative depth structure mainly describes the high-order correlation of the data, or observes the data and obtains the joint probability distribution of the corresponding tags. Unlike the traditional neural network, the generative depth structure can obtain the joint probability distribution of the observation data and the corresponding categories, which can facilitate the estimation of the prior probability and the posterior probability, while the traditional neural network can only estimate the posterior probability. Deep trust networks (DBN) belong to generative depth structure. DBN solves a series of problems existing in traditional BP arithmetic for multifloor neural network, such as large data volume of training sample set, slow convergence speed, and easy to fall into local optimization. DBN consists of a series of restricted Boltzmann machines (RBM) floors. The network structure of RBM is shown in Figure 2.

RBM is made up of two interconnected units: the visible floor and the hidden floor. The following guidelines govern how neurons connect to one another: Although there are connections between neurons in nearby floors, there are none between floors themselves. The visible floor unit is used to define a specific part of the data or a specific feature of the graphics. The feature extraction floor, also known as the visible floor unit, may acquire the correlation between the variables corresponding to the hidden floor unit, as shown in Figure 2. *n*_*v*_, *n*_*h*_ represents the number of neurons contained in the visible floor and the hidden floor, respectively. *v* = (*v*_1_, *v*_2_, *v*_3_, ⋯,*v*_*n*_*v*__)^*T*^ represents the state vector of the visible floor, *v*_*i*_ represents the state of the *i* neuron in the visible floor, *h* = (*h*_1_, *h*_2_, *h*_3_, ⋯,*h*_*n*_*h*__)^*T*^ represents the state vector of the hidden floor, and *h*_*j*_ represents the state of the *j* neuron in the hidden floor. *a* = (*a*_1_, *a*_2_, *a*_3_, ⋯,*a*_*n*_*v*__)^*T*^ ∈ *R*^*n*_*v*_^ represents the offset vector of the visible floor and *a*_*i*_ represents the offset of the *i* neuron in the visible floor. *b* = (*b*_1_, *b*_2_, *b*_3_, ⋯,*b*_*n*_*h*__)^*T*^ ∈ *R*^*n*_*h*_^ represents the offset vector of the hidden floor and *b*_*j*_ represents the offset of the *j* neuron in the hidden floor. *W* = (*w*_*i*,*j*_) ∈ *R*^*n*_*h*_×*n*_*v*_^ represents the weight matrix between the visible floor and the hidden floor, and *w*_*i*,*j*_ represents the connection weight between the *i* neuron in the hidden floor and the *j* neuron in the visible floor. Finding the maximum distribution of the probability of the training samples, or the problem of finding the probability distribution of the maximum possible training samples, is the simplest way to define the RBM training process. The training of RBM can progress into determining the best weight because *W* stands for the weight matrix between the visible floor and the hidden floor, which directly impacts the probability distribution of the training samples. DBN is composed of multiple RBMs combined from bottom to top. The training process is shown in Figure 3.

To ensure that as much feature information as possible can be kept when feature vectors are transferred to various feature spaces, each floor of the RBM network is first trained unsupervised individually, sometimes referred to as pretraining. Second, to train the classifier in a supervised way, a BP network is added to the last floor of the DBN using the feature vector output from the RBM of the previous floor as its input feature vector. The BP network will also fine-tune the complete DBN network and relay the error information to each RBM floor from back to front. This is due to the fact that each RBM network floor only makes sure that its weight is optimal for its own feature vector mapping and not the feature mapping of the entire DBN network. The disadvantages of BP networks, such as lengthy training times and settling into local optimal solutions as a result of random initialization of weight parameters, can be solved by using RBM to train the model in DBN networks.

#### 3.2.2. Discriminant Depth Structure

Discriminant depth structure's primary purposes are to discern patterns and explain the posterior probability distribution of data. Due to its multilevel network structure, CNN is able to minimize preprocessed input, simplify the model structure by employing shared weights, and reduce the number of parameters by depending on spatial correlations.

1. The floor of convolution CNN first applies the convolution kernel and convolution floor biassing to the input graphics. Calculus's fundamental mathematical formulation for convolution is

(2) $$\begin{array}{c} S\left(t\right)=\int x\left(t-a\right)w\left(a\right)\text{da}. \end{array}$$

The discrete form of formula (2) is expressed as

(3) $$\begin{array}{c} s\left(t\right)=\underset{a}{\sum }x\left(t-a\right)w\left(a\right). \end{array}$$

If expressed in matrix form, it is expressed as

(4) $$\begin{array}{c} s\left(t\right)=\left(X*W\right)\left(t\right). \end{array}$$

In equation (4), ∗ denotes convolution operation.

The mathematical formulation of CNN network's two-dimensional convolution operation is

(5) $$\begin{array}{c} s\left(i,j\right)=\left(X*W\right)\left(i,j\right)=\underset{m}{\sum }\underset{n}{\sum }x\left(i+m,j+n\right)w\left(m,n\right). \end{array}$$

In equation (5), *W* is the convolution kernel in the convolution floor, and *X* is the input data. If *X* is a two-dimensional input matrix, *W* is also a two-dimensional matrix. If *X* is a multidimensional vector, *W* is also a multidimensional vector. The convolution kernel matrix and the elements at various points of the various local matrices of the input graphics are multiplied and added by the convolution floor when it performs convolution operation on those visuals. The neural network must make sure that each neuron in the network can adapt to complicated nonlinear operations, however, and since this operation is linear, this necessitates the insertion of nonlinear elements, namely the activation function. Its nonlinearity, continuous differentiability, monotonicity, and approximative linearity at the origin are all positive mathematical properties of the activation function. The sigmoid, tanh, and relu functions are the most often utilized activation functions.

The convolution floor of the CNN model contains numerous convolution kernels. The feature map of the input visuals can be obtained by each convolution kernel following the convolution process, and these feature maps share the same weight matrix and offset vector. The typical graphics are output once the convolution result has been averaged.

(6) $$\begin{array}{c} {\text{Y}}_{j}=\frac{\left(\sum_{i=0}^{N}W_{j}\times X_{i}\right.}{N} \end{array}$$

(2) The pooled floor graphics is sent to the pooled floor for aggregation statistics after the feature map of the graphics is obtained through the convolution floor. The pooling floor is mainly responsible for the aggregation of feature graphics
(3) Full connection floor. The full connection floor is the “Classifier” of the entire CNN network. Its main function is to map the feature representation after convolution and pooling operations to the corresponding sample label space

#### 3.2.3. Hybrid Depth Structure

The purpose of the mixed depth structure is to distinguish the data. Its learning process includes two parts, i.e., the generative part and the discriminative part. Firstly, the generative depth structure is used to classify the objects, and the network ownership value is optimized in the pretraining stage of the structural model combined with the discriminative depth structure.

## 4. Result Analysis and Discussion

University culture and emotion are derived from the campus life and practical experience of specific people in the campus. Giving product emotion is to consolidate the emotional connection of the audience to the campus life. When the progress and design of cultural and innovative goods in universities meet their functions, they must also materialize the culture and feelings of universities into physical objects, so that they can become campus cultural and innovative goods integrating functions and feelings. In this process, we must find a rich campus culture and emotional tone, and establish an appropriate emotional “situation” to stimulate the audience's consumption desire.

Input the test samples into the network model for testing. The test sample is 10000 campus pictures. During the test, the test samples pass through the same network structure, but the bias parameter *B* vector and the weight parameter *W* matrix in the network are learned by the training part. This chapter selects a group of representative handwritten digital pictures to test the recognition results (including recognition efficiency and recognition accuracy). The results are shown in Table 1.

Comparing the data in Table 1, under the same experimental conditions, the accuracy of the enhanced CNN model on the test set can reach 97.22%. Compared with the traditional CNN model, the accuracy rate has increased from 91.35% to 97.22%, and the recognition efficiency has increased from 83.16 s to 13.45 s. It can be said that the recognition of campus innovative cultural elements is a leap forward.

In order to verify the recognition performance of the enhanced arithmetic, MNIST and petdataset datasets are selected for experiments. The error rate change curves of the enhanced arithmetic (CNN combined with Parzen classifier) and the original arithmetic (CNN combined with softmax classifier) on MNIST and petdataset datasets are shown in Figures 4 and 5. It can be seen from Figure 4 that the enhanced arithmetic uses fewer training times (3000 times) than the original arithmetic (4000 times) when it reaches a lower error recognition rate, and the recognition efficiency is significantly enhanced.

It can be seen from Figure 5 that the enhanced arithmetic uses fewer training times (3000 times) than the original arithmetic (5000 times) when reaching a lower false recognition rate, which significantly enhances the recognition efficiency. It can also be seen from Figures 4 and 5 that as the number of iterations increases, the error recognition rate of the two arithmetic on each dataset continues to decline and finally converges, indicating that the enhanced arithmetic has strong generalization performance.

In order to verify the convergence of the enhanced arithmetic, MNIST and petdataset datasets are selected for experiments. The changes of the convergence curve during the iteration of the enhanced arithmetic and the original arithmetic on MNIST and petdataset are shown in Figure 6.

Because the convergence index of the two groups of arithmetic changes greatly, the convergence curves in the same group are close, and it is difficult to distinguish. Therefore, the previous and later stages of the training process in Figure 6 are, respectively, enlarged. The change of the convergence curve in the previous training process is shown in Figure 7, and the change of the convergence curve in the later training process is shown in Figure 8.

By analyzing Figures 6–8, it can be found that with the increase of the number of iterations (epoch), the convergence index of the enhanced arithmetic and the original arithmetic on the MNIST and petdataset datasets continues to decline, and finally, both reach convergence. But the convergence speed of the enhanced arithmetic is faster and the convergence effect is better than the original arithmetic.

This chapter proposes to use Parzen classifier combined with CNN for graphics recognition. First, CNN is used to automatically learn the graphics features, and then, Parzen classifier is used to classify and recognize the graphics according to the extracted graphics features. Experiments on MNIST and petdataset show that compared with the traditional CNN combined with softmax method, the recognition accuracy of CNN combined with Parzen method is greatly enhanced; Moreover, the number of iterations used to achieve high recognition accuracy is significantly reduced, which saves the running time and enhances the recognition efficiency. Moreover, the enhanced arithmetic has strong generalization performance.

## 5. Conclusions

This article suggests a design strategy for campus cultural inventive commodities that is optimum for both progress and emotional expression research in universities. It first builds a data mining system for the graphics recognition of campus cultural products before concentrating on the issue of DL-based graphics recognition. The accuracy and effectiveness of graphics recognition are proposed to be improved via an improved DL model and arithmetic. The simulation test and analysis are completed in the end. The simulation results demonstrate a certain accuracy for the suggested arithmetic, which is 10.23% greater than the conventional DL arithmetic. This outcome demonstrates in full how well DL can extract data features in the setting of huge data and how robust its data representation capabilities are. Researchers have examined and used DL technology in the disciplines of images, text, voice, and more. The advancement of culture at universities is crucial since humanistic and aesthetic education are given more and more importance. College cultural and creative goods combine culture, beauty, function, and emotion and can help institutions gain more cultural values and money. Universities should pay more attention to the development of cultural and innovative products so that they can eventually make a breakthrough in the creation of their own cultural and inventive products. The choice of materials, the consideration of multifunction, the range of series, and the degree of grade are just a few of the latter design and production stages that still need improvement. Additionally, some things cannot really be made due to a variety of problems. In next research and study, it is envisaged that broader design thinking can be developed.

## Figures and Tables

**Figure 1:** Framework of graphics mining.

**Figure 2:** RBM structure.

**Figure 3:** DBN training process.

**Figure 4:** MNIST error rate change curve.

**Figure 5:** Change curve of petdataset error rate.

**Figure 6:** Convergence curve of MNIST and petdataset.

**Figure 7:** Convergence curve in the early stage of training.

**Figure 8:** Convergence curve at the later stage of training.

**Table 1:** Experimental results of traditional MLP, traditional CNN, and enhanced CNN.

Arithmetic	Network level	Number of iterations	Recognition rate	Training time
Traditional MLP	4	500	93.65	57.95
Traditional CNN	11	500	91.35	83.16
Improve CNN	3	500	97.22	13.45

## Data Availability

The data used to support the findings of this study are available from the corresponding author upon request.
